# Deubiquitination of TNKS1 Regulates Wnt/*β*-Catenin to Affect the Expression of USP25 to Promote the Progression of Glioma

**DOI:** 10.1155/2022/9087190

**Published:** 2022-04-11

**Authors:** Bin Tang, Hai Luo, Shenhao Xie, Chengbing Pan, Jun Fu

**Affiliations:** Department of Neurosurgery, The First Affiliated Hospital of Nanchang University, Nanchang 330006, China

## Abstract

**Objective:**

To explore the regulatory effect of ubiquitin specific protease 25 (USP25) on glioma cell proliferation, migration, invasion, and its underlying mechanism.

**Methods:**

The USP25-overexpressed and USP25-knockdown glioma cells were established on U251 and U87 cells, respectively. Glioma cell proliferation ability was evaluated by CCK-8 assay. Cell apoptosis and cell cycle were determined utilizing flow cytometry. The Transwell assay measured cell invasion with wound healing used for cell migration detection. Western blotting established key protein expression levels in the Wnt/*β*-catenin pathway. The coimmunoprecipitation was used to check Thankyrase 1 (TNKS1) ubiquitination levels.

**Results:**

TNKS1 expression levels were found to be considerably repressed in USP25-knockdown glioma cells and elevated in USP25-overexpressed glioma cells, accompanied by Wnt/*β*-catenin pathway key protein downregulation and upregulation, respectively. Glioma cell invasion, migration, and proliferation activity were dramatically inhibited in USP25-knockdown glioma cells and promoted in USP25-overexpressed glioma cells. TNKS1 ubiquitination level was knowingly increased in USP25-knockdown glioma cells and reduced in USP25-overexpressed glioma cells, suggesting TNKS1 ubiquitination levels were negatively regulated by USP25.

**Conclusion:**

USP25 facilitated glioma cell invasion, migration, and proliferation by regulating Wnt/*β*-catenin through the deubiquitination on TNKS1.

## 1. Introduction

Glioma, accounting for around 80% of central nervous system (CNS) primary malignant tumors, is the most widespread primary malignant intracranial brain tumor. Due to the high recurrence rate, drug resistance, and high mortality, rare progression has been achieved by the current treatments of radiotherapy and chemotherapy. In recent years, novel strategies have been proposed based on targeted molecular therapies. It is critical to conduct in-depth research on the pathological molecular mechanism of glioma and offer a theoretical basis for promising therapeutic targets.

The Wnt/*β*-catenin signaling pathway is a vital part of adult development and homeostasis, and its abnormal regulation is informed to facilitate malignant tumor development and progression [1]. The mutations in *β*-catenin/Wnt or truncation mutation on adenomatous polyposis coli protein (APC) can induce the over activation of the Wnt/*β*-catenin signaling pathway, which further promotes the development of colorectal carcinoma, gastric carcinoma, and hepatoma [2, 3]. Therefore, Wnt/*β*-catenin pathway inhibitor development as a new anticancer therapy will be a major breakthrough in the field of malignant tumors [4, 5]. Thankyrase (TNKS) is initially found to be a regulator of telomere maintenance and facilitates the separation of telomeric repeat binding protein 1 (TRF1) from cell telomere to induce the combination of telomere and telomere, which maintains the telomere at a specific length to participate in malignant tumor development. In the Wnt/*β*-catenin signaling pathway, Axin is glycosylated by TNKS, and the glycosylated Axin induces the ubiquitination of TNKS and the degradation of the proteasome by acting on the ubiquitin E3 ligase RNF146 [6–8]. *β*-Catenin will be downregulated by the stably expressed Axin, which results in the declined transcriptional activity of *β*-catenin. Mariotti et al. [9] reported that the degradation of *β*-catenin could be induced by the inhibition on TNKS (TNKS1 and TNKS2), which further reduced colorectal cancer cell Wnt signaling activity. Therefore, inhibition of TNKS is considered as a novel method for malignant tumor treatment by blocking the Wnt signaling pathway [6, 10, 11].

Deubiquitination is a vital protein stability regulating cellular mechanism [12]. A deubiquitination enzyme, ubiquitin specific protease 25 (USP25), inhibits substrate protein degradation by specifically recognizing the deubiquitination-related substrate proteins, which are vital in maintaining cellular normal function. Though, USP25 regulatory role in glioma remains unclear. Xu et al. [13] found that USP25 directly interacted with TNKS via the C-terminal tail to promote TNKS stabilization and deubiquitination, which further regulates the Wnt/*β*-catenin signaling pathway. USP25 exerts a vital part in human malignant tumor cell proliferation and migration [14, 15]. Therefore, we suspected that USP25 impacts glioma cell development and growth by Wnt/*β*-catenin signaling pathway regulation via mediating TNKS1 ubiquitination.

Therefore, in the present study, we investigated the effect of USP25 on the level of ubiquitination of TNKS1 and on the function and mechanism of glioma cell proliferation, invasion, and migration by interfering with the expression of USP25 in human glioma cells U87 and U251.

## 2. Methods

### 2.1. Cells and Treatments

U251 (Art. No. CL-0237) and U87 cells (Art. No. CL-0238) were bought from Procell (Wuhan, China). The cells were cultured in DMEM completed medium (Gibco, USA) supplemented with 10% fetal bovine serum (FBS; Gibco, USA) under the condition of 5% CO_2_ and 37°C.

### 2.2. Cell Transfection

To knockdown or overexpress USP25 in glioma cells, USP25-siRNAs, and its control (siRNA NC), USP25 overexpression vector pcDNA3.1-USP25 (OE) and control pcDNA3.1-NC (OE NC) were designed and synthesized by General Biol. Inc. (Anhui, China). The above interfering fragments or vectors were transfected into U87 and U251 cells, respectively, using Lipofectamine 3000 (Invitrogen, California, USA). After 48 h of transfection, the cells were collected for subsequent assays. The sequences for siRNAs were illustrated in Table 1.

### 2.3. Western Blotting

Following extracting proteins from tissues and cells, quantification was performed on proteins, which were loaded onto 12% SDS-PAGE. Following separating for 1.5 h, proteins were transferred onto the PVDF membrane (Takara, Tokyo, Japan) and using 5% skim milk for blocking, followed by adding the primary antibody against TNKS1 (cat. ab83978, Abcam, Cambridge, UK), Cyclin D1 (cat. ab226977, Abcam, Cambridge, UK), C-myc (cat. ab17355, Abcam, Cambridge, UK), *β*-catenin (cat. DF6794, Affintiy, Melbourne, Australian), phosphorylation-*β*-catenin (p-*β*-catenin; cat. AF3266, Affintiy, Melbourne, Australian), and GAPDH (1 : 1000, Affintiy, Melbourne, Australian), respectively. After incubation with the secondary antibody (1 : 2000, Affintiy, Melbourne, Australian) for 1.5 h, the membrane was hatched with the enhanced chemiluminescence (ECL) solution (RJ239676, Thermo Fisher, USA), followed by the ImageJ software quantification.

### 2.4. Quantitative Real-Time PCR (RT-qPCR)

Cell total RNA isolation was conducted with the TRIzol© reagent (Invitrogen. California, USA), then transcribed into cDNAs utilizing the TaqMan miRNA reverse transcription kit (Invitrogen. California, USA). The ABI 7900 real-time PCR machine was applied to conduct the PCR reaction using the SYBR® Green Real-time PCR Master Mix (Roche Diagnostics, Basel, Switzerland). The 2^−*ΔΔ*Ct^ method was utilized to determine the normalization of gene expression completed with *β*-actin.  Table 2 illustrates primer sequences.

### 2.5. CCK8 Assay

In brief, after digesting cells using 0.25% pancreatin, cells (5 × 10^3^/well) were planted on 96-well plates for 24-hour incubation. The culturing medium supplemented with 10% CCK-8 solution (KGA317, KeyGEN BioTECH, Jiangsu, China) was then replaced. Finally, after 2 h, 570 nm absorbance was quantified with the use of the microplate reader (Molecular Devices, California, USA).

### 2.6. Wound Healing Assay

After seeding cells onto 6-well plates to 80% confluence, the sterile plastic pipette tips were utilized to scrap the cell monolayer, followed by twice washes using the serum-free medium. After different strategies for 24 hours, images of the wound closure were taken using the inverted microscope (Laird, Missouri, USA).

### 2.7. Transwell Assay

Cells (5 × 10^4^/well) were planted on the insert upper chamber (Corning, Cambridge, USA). Medium comprised of 1% FBS was included in the lower chamber before 37°C incubation for 24 h. Then, the membrane upper surface was eliminated, and 0.1% crystal violet was utilized to stain lower chamber cells. Lastly, images were taken using the inverted microscope (Laird, Missouri, USA).

### 2.8. Coimmunoprecipitation (Co-IP) Assay

Prechilled phosphate-buffered saline (PBS) was used to wash the transfected cells and lysed. After centrifugation, 50 *μ*l supernatant was used as Input. Boiling of the cell lysates was done for 15 min before dilution with 1 : 10 ratio deubiquitination inhibitors and protease inhibitors in NP-40 lysis buffer. Lastly, protein A/G beads (IP05, Millipore, USA) and antibodies or control lgG were utilized to perform immunoprecipitation at 4°C for 4 h. After washing the beads three times with 1 ml of lysis buffer, the immuno-complexes underwent Western blot assay.

### 2.9. Statistical Analysis

Data gained were presented as mean ± standard deviation (SD) with the GraphPad software used for analyzing. Disparities between the two groups were analyzed with the application of the Student's *t*-test. Disparities between groups were evaluated with the one-way ANOVA method. *P* < 0.05 was deemed a considerable difference in this study.

## 3. Results

### 3.1. The USP25-Overexpressed and USP25-Knockdown Glioma Cells Were Established

As shown in Figures 1(a)–1(d), RT-qPCR was used to examine the transfection efficiency of USP25 interference or overexpression in glioma cells. In U251 and U87 cells, compared with the siRNA-NC group, USP25 expression levels were significantly repressed by the transfection with siNRA-1, siNRA-2, or siNRA-3 (*P* < 0.05). Compared to the USP25 OE NC group (pcDNA3.1-NC transfected cells), USP25 was dramatically upregulated in the USP25 OE (pcDNA3.1-USP25 transfected cells) group (*P* < 0.05). Among the three siRNAs, USP25 expression in glioma cells transfected with siRNA-2 was the lowest. Therefore, siRNA-2 was chosen to knockdown USP25 in glioma cells in the subsequent experiments.

### 3.2. USP25 Overexpression Increased the TNKS1 Expression in the Glioma Cells

In Figure 2, it can be seen that in both U87 and U251 cells, when contrasted against the siRNA NC group, TNKS1 expression was found significantly downregulated by the transfection of siRNA-USP25 (*P* < 0.05). On the contrary, compared to the OE NC group, a significantly higher expression of TNKS1 was detected in pcDNA3.1-USP25 transfected glioma cells (*P* < 0.05). These results revealed that TNKS1 expression was positively regulated by USP25 in the glioma cells.

### 3.3. USP25 Facilitated U251 and U87 Cell Proliferation

CCK-8 assay was employed for proliferation ability determination of U251 and U87 cells following different treatments. As indicated in Figure 3, contrasted to the siRNA NC group, significantly declined cell viability was observed in U251 or U87 cells transfected with siRNA-USP25 (*P* < 0.05). On the contrary, compared to the OE NC group, cell viability was dramatically elevated in glioma cells transfected with pcDNA3.1-USP25 (*P* < 0.05). Findings gained collectively proposed that proliferation of glioma cells was significantly facilitated by USP25.

### 3.4. USP25 Induced the Migration of U251 and U87 Cells

The wound healing assay was employed to assess glioma cell migration ability.  Figure 4 shows that in comparison to the siRNA NC group, the migration ability in siRNA-USP25 transfected U251 cells or U87 cells was significantly decreased (*P* < 0.05). On the contrary, compared with OE NC, the migration ability was significantly increased after USP25 overexpression (*P* < 0.05), indicating that glioma cell migration ability was greatly facilitated by USP25.

### 3.5. USP25 Accelerated U251 and U87 Cell Invasion

The invasion ability of glioma cells was determined by the Transwell assay.  Figure 5 shows that compared to the siRNA NC group, considerably less invaded cells were observed in U251 cells or U87 cells transfected with siRNA-USP25 (*P* < 0.05). Compared to the OE NC group, invaded cell numbers dramatically declined in pcDNA3.1-USP25 transfected glioma cells (*P* < 0.05), revealing that glioma cell invasion ability was greatly facilitated by USP25.

### 3.6. USP25 Activated the Wnt/*β*-Catenin Pathway in U87 and U251 Cells

Figures 6(a) and 6(b) show that contrasted to the siRNA NC group, Cyclin D1, p-*β*-catenin, *β*-catenin, and c-myc levels expressed were greatly repressed in siRNA-USP25 transfected U251 cells or U87 cells (*P* < 0.05). However, after overexpression of USP25, all the above proteins were significantly upregulated (*P* < 0.05). This outcome indicates that USP25 activates the Wnt/*β*-catenin pathway in glioma cells.

### 3.7. USP25 Inhibited the Level of TNKS1 Ubiquitination in U251 Cells

Ubiquitination levels in U251 cells were evaluated by the Co-IP assay.  Figure 7 shows that in contrast with the input, TNKS1 was considerably enriched after Co-IP, indicating that TNKS1 was successfully pulled down in U251 cells. Compared to the siRNA NC group, the ubiquitination level in siRNA-USP25 transfected U251 cells was substantially promoted. In comparison with the OE NC group, pcDNA3.1-USP25 transfected U251 cell ubiquitination levels greatly declined. These data showed that TNKS1 deubiquitination in U251 cells was significantly induced by USP25.

## 4. Discussion

Although novel techniques have been applied in the chemotherapy, radiotherapy, and surgery for glioma treatment in recent years, patient's survival continues to be poor due to the high degree of malignancy in glioma and the blurred interface between the lesion site and surrounding normal tissues.

High expression of TNKS1 in multiple types of malignant tumors has been reported, involving the digestive tract, bladder, breast, and lung cancers [16–21]. Our previous research revealed that compared to normal brain tissues, TNKS1 was considerably upregulated in glioma tissues, and TNKS1 levels expressed were closely associated with the pathological grading of glioma [22]. In malignant tumor occurrence and development, Wnt signaling pathway is found abnormally activated and regulates the progression of proliferation, migration, and invasion by coordinating or antagonizing with other signaling pathways [23]. Earlier studies of our own found that TNKS1 and *β*-catenin were dramatically upregulated in glioma tissues when matched against normal brain tissue, implying that Wnt/*β*-catenin pathway may be a vital part of glioma as a classical signaling pathway positive regulator [24]. Lately, reports have stated that in colorectal cancer with classical APC gene mutation, the protein stability of Axin could be enhanced by inhibiting the activity of TNKS1, which further induces *β*-catenin degradation and Wnt signaling pathway inhibition [9]. Feng et al. [25] claimed that TNKS1 could regulate the Wnt/*β*-catenin signaling pathway positively during mouse embryonic development progression, indicating that downregulation of TNKS1 might suppress the Wnt/*β*-catenin signaling pathway in glioma cells. Our prior data discovered that TNKS1 could facilitate the *β*-catenin nuclear transport, which further activates downstream target gene transcription expression, including Cyclin D1 and c-myc, to stimulate glioma cell proliferation and invasion [26].

USP25 is closely linked with malignant tumors, immune responses, and inflammation. For instance, USP25 is related to the endoplasmic reticulum-associated degradation, and the processing of amyloid precursor protein could be regulated by the acute ER stress-mediated ubiquitin dependent degradation [27, 28]. USP25 is an interleukin-17 signaling and inflammation negative regulator by removing TRAF3, TRAF5, and TRAF6 [29]. USP25 has been informed to be vastly expressed in human breast cancer tissues with a 3-fold change [30], and USP25 may be a human lung cancer tumor suppressor [31]. The research on human non-small-cell lung cancer revealed that tumor cell metastasis and invasion were repressed by miR-220c through targeting USP25 [14], which was constant with present study outcomes that the invasion, migration, and proliferation of U251 and U87 glioma cells could be inhibited and promoted by the knockdown and overexpression of USP25, respectively.

Recent studies have shown that Wnt signaling is positively regulated by USP25 mediating TNKS deubiquitination, while the degradation of TNKS1 could be facilitated by USP25, which contributes to Axin stabilization and the inactivation of Wnt/*β*-catenin signaling. In addition, the C-terminus of USP25 is found to interact with anchor protein repeats of TNKS1 directly, and X-ray crystal structure determination further characterizes the TNKS1 and USP25 interaction [13]. In the current study, P-*β*-catenin, Cyclin D1, *β*-catenin, and C-myc levels expressed in the Wnt pathway were positively regulated by USP25 in U251 and U87 glioma cells. Additionally, in U251 cells, TNKS1 ubiquitin level in the USP25-knockdown group was amplified, while TNKS ubiquitin levels in the USP25 overexpression group were considerably decreased, implying that TNKS1 ubiquitin levels in U251 cells were negatively regulated by USP25. The role of USP25-mediated ubiquitination of TNKS1 in regulating the Wnt pathway in glioma cells was further verified. To date, no therapeutic role has been found regarding USP25 in glioma. In contrast, this study provides a direct research basis for USP25 as a therapeutic target in glioma and its mechanism with TNKS1, and USP25 will become another significant discovery in glioma treatment.

## 5. Conclusion

All in all, the data gained revealed that USP25 facilitated glioma cell invasion, migration, and proliferation by Wnt/*β*-catenin regulation through the deubiquitination on TNKS1.

## Figures and Tables

**Figure 1:** RT-qPCR determined USP25 transfection efficiency in the U87 and U251 cells. USP25-siRNAs (siRNA-1, -2, -3) and control (siRNA NC) and USP25 overexpression vector pcDNA3.1-USP25 (OE) and control pcDNA3.1-NC (OE NC) were transfected into U87 (a, b) and U251 cells (c, d). Control, no treatment. ^∗^*P* < 0.05 vs. Control group; #*P* < 0.05 vs. siRNA NC or USP25 OE NC group. The experiment was repeated three times.

**Figure 2:** USP25 overexpression increased the TNKS1 expression in the glioma cells. The TNKS1 expression in the U87 and U251 cells was measured by Western blotting. ^∗^*P* < 0.05 vs. Control group; #*P* < 0.05 vs. siRNA NC group; *ΔP* < 0.05 vs. OE NC group.

**Figure 3:** USP25 promoted U251 and U87 cell proliferation. CCK-8 assay was used to measure U87 and U251 cell proliferation after transfection with USP25 siRNA or overexpression vector. ^∗^*P* < 0.05 vs. Control group; #*P* < 0.05 vs. siRNA NC group; *ΔP* < 0.05 vs. OE NC group. The experiment was repeated three times.

**Figure 4:** USP25 induced the migration of U251 and U87 cells. Wound healing assay was applied to determine the migration ability of U87 and U251 cells after transfection with USP25 siRNA or overexpression vector. ^∗^*P* < 0.05 vs. Control group; #*P* < 0.05 vs. siRNA NC group; *ΔP* < 0.05 vs. OE NC group.

**Figure 5:** USP25 accelerated U251 and U87 cell invasion. U87 and U251 cell invasion was detected utilizing Transwell assay after transfection with USP25 siRNA or overexpression vector. ^∗^*P* < 0.05 vs. Control group; #*P* < 0.05 vs. siRNA NC group; *ΔP* < 0.05 vs. OE NC group.

**Figure 6:** USP25 activated the Wnt/*β*-catenin pathway. The expression of Cyclin D1, p-*β*-catenin, *β*-catenin, and c-myc in U87 (a) and U251 (b) cells was detected by Western blotting. ^∗^*P* < 0.05 vs. Control group; #*P* < 0.05 vs. siRNA NC group; *ΔP* < 0.05 vs. OE NC group.

**Figure 7:** USP25 inhibited the level of TNKS1 ubiquitination. The ubiquitination level of TNKS1 was determined by the coimmunoprecipitation assay.

**Table 1:** siRNA sequences.

siRNAs	Sequences (5′-3′)
USP25-siRNA-1	GUAAUGGAAACUUGGAAUUTT
	AUUCCAAGUUUCCAUUACTT
USP25-siRNA-2	CCAUUAGCAGAGUUCUUGATT
	CAAGAACUCUGCUAAUGGTT
USP25-siRNA-3	GUUAUUCAGUCAUUAUUUATT
	UAAAUAAUGACUGAAUAACTT
NC	UUCUCCGAACGUGUCACGUTT
	ACGUGACACGUUCGGAGA ATT

**Table 2:** The sequences of primers in RT-qPCR assay.

Primers	Sequences (5′-3′)
USP25	Forward: ACCCCACCAGAAACCGATTAT
USP25	Reverse: ATAATCCTGATGCCACTCCTCATA
*β*-Actin	Forward: TGGCACCCAGCACAATGAA
*β*-Actin	Reverse: CTAAGTCATAGTCCGCCTAGAAGCA

## Data Availability

The data used to support the findings of this study are included within the article. Further inquiries can be directed to the corresponding author.
